# Automated Atrial Fibrillation Detection Based on Feature Fusion Using Discriminant Canonical Correlation Analysis

**DOI:** 10.1155/2021/6691177

**Published:** 2021-04-08

**Authors:** Jingjing Shi, Chao Chen, Hui Liu, Yinglong Wang, Minglei Shu, Qing Zhu

**Affiliations:** ^1^Shandong Artificial Intelligence Institute, Qilu University of Technology (Shandong Academy of Sciences), China; ^2^Qilu Hospital of Shandong University, China

## Abstract

Atrial fibrillation (AF) is one of the most common cardiovascular diseases, with a high disability rate and mortality rate. The early detection and treatment of atrial fibrillation have great clinical significance. In this paper, a multiple feature fusion is proposed to screen out AF recordings from single lead short electrocardiogram (ECG) recordings. The proposed method uses discriminant canonical correlation analysis (DCCA) feature fusion. It fully takes intraclass correlation and interclass correlation into consideration and solves the problem of computation and information redundancy with simple series or parallel feature fusion. The DCCA integrates traditional features extracted by expert knowledge and deep learning features extracted by the residual network and gated recurrent unit network to improve the low accuracy of a single feature. Based on the Cardiology Challenge 2017 dataset, the experiments are designed to verify the effectiveness of the proposed algorithm. In the experiments, the F1 index can reach 88%. The accuracy, sensitivity, and specificity are 91.7%, 90.4%, and 93.2%, respectively.

## 1. Introduction

Atrial fibrillation (AF) is the most common persistent cardiovascular disease, which can easily lead to strokes, hemiplegia, and other diseases, seriously threatening patients' health; thus, timely diagnosis and treatment are necessary. However, owing to the shortage of medical resources and the single model of doctor diagnosis, it becomes urgent to improve automatic detection technology. Automatic detection of cardiac rhythm is a meaningful and important issue in different age groups, including adults [1] and fetuses [2]. Computational techniques and deep learning methods detecting various types of arrhythmia have been widely developed to analyse ECG signals and are strong candidates to help clinical advances by providing a better understanding of medical challenges [3, 4]. With the development of medicine, people have gained more understanding of the physiological mechanism of atrial fibrillation, but further research is still needed [5]. Physiologically, the occurrence of atrial fibrillation is due to irregular atrial contraction, which is reflected in the electrocardiogram: P waves disappear, irregular fibrillation waves (f waves) of different sizes and shapes appear [6, 7], and there is a severe irregularity of the RR interval.

The detection of atrial fibrillation signals is mainly divided into four parts, including data preprocessing, feature extraction, feature selection, and classification. Among them, feature extraction directly affects the accuracy and efficiency of atrial fibrillation signal classification. Commonly used feature extraction in the literature usually falls into two categories, traditional feature extraction and feature extraction based on deep learning methods. Traditional feature extraction methods are generally divided into three categories. The first is to extract the statistical characteristics of ECG signals, that is, use the statistical data to summarize a series of ECG data. Typical statistics include mean, maximum, minimum, variance, skewness, kurtosis, count, and percentage. Kaya et al. [8] calculated the statistical and time characteristics of a heartbeat, such as skewness, kurtosis, standard, deviation, and average, and they used the best feature reduction and classification methods, the highest classification accuracy, sensitivity, and specificity rates of 99.30%, 98.84%, and 98.40%, respectively. Athif et al. [9] extracted statistical and morphological features and then used a support vector machine classifier to classify records into three categories: “normal,” “AF,” and “other.” The algorithm has a sensitivity of 77.5%, a specificity of 97.9%, and an accuracy of 96.1% in the “Computing in Cardiology Challenge 2017” database. The second is signal processing, which is to transform the ECG data from the time domain to the frequency domain or other domains through discrete Fourier transform, discrete wavelet transform, and other methods. Yin et al. [10] proposed a multidomain ECG feature extraction method. The RR intervals were extracted as time domain feature. The fifth-order approximate coefficients of wavelet decomposition are used to represent the frequency domain features. In addition, the sample entropy values of six wavelet coefficients are used as nonlinear characteristics. These three features were fed to a classifier for automated diagnosis. The average accuracy of the SVM classifier in the MIT-BIH arrhythmia database was 99.70%. The third is to directly extract the time domain or morphological features of ECG signals, including RR interval, QRS wave width, and PR interval. Dash et al. [11] used a statistical method to evaluate the complexity, randomness, and variability of the RR interval. Verification by the MIT-BIH atrial fibrillation database shows the sensitivity is 94.4%, and the specificity is 95.1%. Zabihi et al. [12] adopted time-frequency, phase space, tuples, and other characteristics in multiple fields and used a random forest classifier for feature selection. F1 was 82.6% on the PhysioNet Challenge 2017 atrial fibrillation competition database. Deep learning feature extraction and classification include convolutional neural work (CNN) [13, 14] and long and short memory networks (LSTM) [15, 16] as well as their variants [17, 18]. Warrick and Homsi [19] combined convolutional neural networks and long short-term memory networks (LSTM) and used pooling, step size, and normalization techniques to improve its accuracy. The network predicts a classification every 18 and then selects the final prediction for classification. The total F1 on the PhysioNet Challenge 2017 dataset is 80%.

With the rapid development of deep learning, the advantages of feature-level fusion have become more and more obvious. In recent years, some researchers have used feature fusion for ECG signal detection. Smoleń [20] first used a sequential Recurrent Neural Network (RNN) classifier to get the probabilities for each class and then combined the probabilities with hand-designed features. Finally, F1 is 79% in PhysioNet Challenge 2017 (CinC 2017). Chu et al. [21] proposed a new method for arrhythmia classification based on multilead ECG signals; the core of the design is to fuse two types of deep learning features with some common traditional features and then use a support vector machine (SVM) classifier to classify the feature vectors, and according to the AAMI standard, the accuracy on the 12-lead INCAET dataset is 88.565%. Ghiasi et al. [22] proposed two different classification methods, of which the first is a feature-based method, and the second adopts a deep neural network. Finally, they used the decision table to combine the output results of the two methods and divided all records into three categories. The proposed method is evaluated using a scoring function from the 2017 PhysioNet/CinC Challenge and achieved an overall score of 80% and 71% on the training dataset and hidden test dataset.

This paper presents a robust method capable of detecting AF from single short ECG lead recording. Here are the four main contributions of this paper: (1) novel combination of deep learning and the traditional features; (2) proposed an improved residual network and gated recurrent unit network, which extracted deep learning features in spatial and time series; (3) performing ECG feature fusion used discriminant canonical correlation analysis; and (4) achieving superior classification results compared to the above-cited method of the same database [23–27].

The structure of this paper is as follows: Section 2 introduces the feature extraction method, Section 3 presents the feature fusion method, Section 4 the performance metrics, Section 5 the experimental results and analysis, and Section 6 the summary.

## 2. Feature Extraction

This section mainly introduces deep learning feature extraction methods and traditional feature extraction methods based on expert knowledge.

### 2.1. Dataset

This article uses a large dataset released by the PhysioNet/CinC Challenge in 2017, which contains 8528 single-lead ECG records [28]. Each ECG record in the dataset is collected from an individual. Compared to most of the researches based on the relatively simple dataset, such dataset is of higher research significance. These records are collected by AliveCor equipment. The dataset consists of single-lead ECGs of 8528 subjects of different lengths (about 23,878 heartbeats). The categories include normal rhythm, atrial fibrillation rhythm, other rhythms, and noise. The data duration is 9-60 s.  Table 1 shows the details of the database.

### 2.2. Data Preprocessing

#### 2.2.1. Denoising and Padding

The Butterworth band-pass filter is used to denoise the original ECG. The frequency response of the Butterworth filter is maximally flat (i.e., has no ripples) in the passband and rolls off towards zero in the stopband [29]. The attenuation of the first-order filter is 6 dB per octave, and the attenuation rate of the sixth-order Butterworth filter is 36 dB per octave. Since the frequency range of the ECG signal is mainly concentrated in 0.5 Hz~45 Hz, the blocking frequency is set to 45 Hz here, and the frequency signal output above 45 Hz will be attenuated. Because the convolutional neural network requires the input data to have the same size, but the length of the electrical signal in the center of the dataset is 9 seconds to 61 seconds, the ECG signal should be padded with zeros to adapt to the model.

#### 2.2.2. Sample Balancing

Due to the uneven number of samples in the database, the number of normal rhythms and other rhythm samples is large, namely, 5076 and 2415, respectively, while the number of atrial fibrillation rhythms and noise samples is small, 758 and 279, respectively, which easily affect the performance of model training and overfitting occurs. In this paper, class_weight is used to balance the sample and it provides weights for each output class. The weight of normal and other signals is very small, while the weight of atrial fibrillation and noise signal is much bigger. The class_weight method uses balance, and its weight calculation method: n_samples/(n_classes ∗ np.bincount(y)), where n_classes = 4, np.bincount(y) is the total number of samples for a certain class, and n_sample is the total number of samples, which is 8528. After calculation, the weight of normal ECG recording is 0.42, the weight of the atrial fibrillation signal is 2.81, the other weights are 0.88, and the weight of noise is 7.64.

### 2.3. Deep Learning Feature Extraction

This paper adopts residual network and gated recurrent unit for deep learning network feature extraction, which can not only reduce the depth of the network and effectively prevent overfitting but also extract the timing characteristics of the signal while extracting their spatial characteristics. The specific network structure is shown in Figure 1.

To deal with the degradation of neural networks, the method of establishing identity mapping with residual structure simplifies the multilayer network into a shallower network. According to the characteristics of the residual network, a one-dimensional residual network suitable for processing atrial fibrillation signals is designed. The residual network consists of six residual convolution blocks. In the first two residual blocks, the filter is 16. The residual ConvBlock is composed of four convolution blocks and a one-dimensional average pooling layer. Each convolution block contains a one-dimensional convolution with a step length of 1, a batch normalization, a linear unit with leakage correction, and a spatial random loss. The active layer is finally followed by a one-dimensional average pooling layer, the commonly used batch normalization (BN), LeakyRelu, and SpatialDropout. The spatial random activation function prevents overfitting, which is more conducive to promoting independence between feature maps than dropout. The number of filters in every two residual blocks is doubled, and the convolution step length in each convolution block is 1. The data obtained through the residual network is input into the gated recurrent unit network, and the number of neurons is set to 32; finally, the output of the last hidden layer is extracted as the deep learning feature.

### 2.4. Traditional Feature Extraction

In fact, the ECG signal is used as input to extract relevant statistical features. First, the multilead differential electrocardiogram summation absolute value and adaptive threshold real-time detection algorithm [30] are used to detect QRS points. Taking A0003 in the dataset as an example, the corresponding waveform and the marked R wave are shown in Figure 2.

After the R wave is detected, the RR interval is calculated based on the R wave, and the RR interval is calculated as follows:

(1) $$\begin{array}{c} \text{RRI}=\frac{R_{\text{peaks}}\left(n+1\right)-R_{\text{peaks}}\left(n\right)}{f_{s}}. \end{array}$$

*R*_peaks_(*n*) is the position of the *n*th *R* peak in the sample, and *f*_*s*_ is the sample rate. According to the RR interval and the traditional features of the ECG signal computed by QRS wave, these features are outputs as a feature vector. The RR interval and P wave are shown in Figure 3 [31].

#### 2.4.1. RR Interval Feature

The statistical characteristics of RR intervals include standard deviation and variance, maximum RR interval, minimum RR interval, average RR interval, pNN50 (the proportion of the number of RR intervals in the ECG sequence whose RR interval difference is greater than 50 ms in all RR intervals), RMSSD (root mean square of the difference between the RR intervals), SDSD (standard deviation of the difference between the RR intervals), and the mean, variance, skewness, and kurtosis of each of the RR intervals divided into six segments.

#### 2.4.2. P Wave Feature

The statistical characteristics of the P wave include the mean, variance, skewness, kurtosis, sample entropy, and sample entropy coefficient, and the P wave is divided into the average value, variance, and skewness of each of the six segments.

#### 2.4.3. Signal Procession Feature

In order to extract the features of the ECG signal more comprehensively, we also extract the signal features based on the medical field and the frequency domain. These features first transform ECG data from time domain into frequency domain; then, frequency-related features are extracted. In the presented paper, the periodogram power spectral density (PSD) and energy spectral density are calculated. PSD is calculated using Fast Fourier Transform (FFT). After the transformation, energy within a specific range (band) is obtained. The chosen bands are between 5 frequencies: 0.1, 6, 12, 20, and 30 Hz. Another four features compute the variation based on QRS [1], compute the sample entropy (SampleEn) [2], compute the coefficient of variation and density histograms (CDF) [3], compute the thresholding on the median absolute deviation (MAD) [4], and compute the heart rate variability (variability).

## 3. Feature Fusion

### 3.1. Feature Fusion Based on Feature Concatenation

Based on expert knowledge, this model performs time domain and frequency domain feature extraction on the denoised ECG signal to obtain feature vectors. It uses a convolution residual network and gated recurrent unit to form a deep learning network, and input data filled ECG signal deep learning network to obtain deep feature vectors.

The two feature vectors obtained are fused into one feature vector in series and input into the classifier composed of the fully connected layers to classify ECG signals, as shown in Figures 4 and 5. This method is simple and but highly applicable. Compared with single feature extraction and classification [33], this method has improved accuracy [32]. However, since the method of fusion features is simple and rough, there are problems of redundancy and a large amount of calculation [34].

### 3.2. Feature Fusion Based on DCCA

In view of the shortcomings of the above-mentioned concatenation method, this section uses discriminant canonical correlation analysis (DCCA) [35] for feature fusion. DCCA is an improvement in canonical correlation analysis (CCA) [36]. The CCA feature fusion process does not consider the class structure. The DCCA method can not only optimize the correlation among the four types of samples but also minimize the correlation among the features of different types of samples. The proposed DCCA feature fusion method is shown in Figure 6.

In this paper, the discriminant canonical correlation analysis (DCCA) method is used for deep learning feature and traditional feature fusion, the preprocessed ECG signals are extracted separately to obtain two feature vectors, and then the DCCA method is used for feature fusion. The specific implementation is divided into four steps as follows:

1. Find a set of projection direction *w*_*x*_ and *w*_*y*_ to achieve the maximum correlation among the features of samples of the same type and the minimum correlation among the features of different types of samples. Mathematically, DCCA is to maximize the correlation coefficient. The formula is as follows:

(2) $$\begin{array}{c} J_{\text{d}}\left(w_{x},w_{y}\right)=\frac{w_{x}^{T}{\tilde{S}}_{xy}w_{y}}{\sqrt{w_{x}^{T}S_{xx}w_{x}w_{y}^{T}S_{yy}w_{y}}}, \end{array}$$

where ${\tilde{S}}_{xy}=S_{w}-\eta S_{b}$ (adjustable parameter > 0), *S*_*w*_ is the intraclass correlation matrix, *S*_*b*_ is the interclass correlation matrix, adjustable parameters *η* measure the relativity of the intraclass correlation and the interclass correlation of the sample characteristics, and the definitions of intraclass correlation and interclass correlation are shown in Figure 7

(2) Calculate the intraclass correlation matrix *S*_*w*_ and the interclass correlation matrix *S*_*b*_, and set the processed sample set as

(3) $$\begin{array}{c} X=\left[x_{1}^{\left(1\right)},\cdots x_{n1}^{\left(1\right)},\cdots ,x_{1}^{\left(c\right)},x_{nc}^{\left(1\right)}\right]\in R^{p\times n},\\ Y=\left[y_{1}^{\left(1\right)},\cdots ,y_{n1}^{\left(1\right)},\cdots ,y_{1}^{\left(c\right)},y_{nc}^{\left(1\right)}\right]\in R^{q\times n}. \end{array}$$

Then, the intraclass correlation matrix and the interclass correlation matrix are, respectively, shown as

(4) $$\begin{array}{c} S_{w}=\overset{c}{\underset{i=1}{\sum }}\overset{n_{i}}{\underset{k=1}{\sum }}\overset{n_{i}}{\underset{l=1}{\sum }}x_{k}^{\left(i\right)}y_{l}^{\left(i\right)T}=XDY^{T}, \end{array}$$

where *D* is a block diagonal matrix, which is also a positive semidefinite matrix. The difference between the interclass correlation matrix and the intraclass correlation matrix is just a negative sign [37]

(3) Solve the eigenvalues and eigenvectors. The optimization problem of DCCA can be transformed into

(5) $$\begin{array}{c} \max w_{x}^{T}S_{w}w_{y}\text{ s}.\text{t}.w_{x}^{T}S_{xx}w_{x}=w_{y}^{T}S_{yy}w_{y}=1. \end{array}$$

Use the Lagrangian multiplier method to solve the above optimization problem turning the above problem into a problem of finding characteristic roots and characteristic vectors.

(6) $$\begin{array}{c} S_{w}S_{yy}^{-1}{\left(S_{w}\right)}^{T}w_{x}=\lambda^{2}S_{xx}w_{x},\\ {\left(S_{w}\right)}^{T}S_{xx}^{-1}S_{w}w_{y}=\lambda^{2}S_{yy}w_{y}. \end{array}$$

The eigenvector {*w*_*x*_, *w*_*y*_}_1_^*d*^ corresponds to the first d generalized eigenvalues, and the *λ*_1_ ≥ *λ*_2_ ≥ *λ*_*d*_

(4) For each pair of samples (*x*, *y*), fusion is performed according to the tandem method. The block diagram of feature fusion using the DCCA algorithm is shown in Figure 8

## 4. Performance Metrics

In order to optimize the atrial fibrillation detection model, a large number of experiments are carried out using a single-lead ECG dataset. The experiment in this article is to train on a server equipped with Tesla V100-SXM2 GPU and Ubuntu 16.04 operating system, and its dynamic memory of the computer is 32480MiB.

In this paper, normal F1 score, atrial fibrillation F1 score, other F1 score, and the average value of three categories of F1 score are four metrics for evaluating the classification performance of the experiments. The definition of these four metrics can be defined as

(7) $$\begin{array}{c} F_{1a}=\frac{2\times A_{a}}{\sum A+\sum a}, \end{array}$$

where *A* is the total number of signals identified as atrial fibrillation by the algorithm, *A*_*a*_ is the number of signals correctly classified as atrial fibrillation by the algorithm, and *a* is the total number of atrial fibrillation signals.

(8) $$\begin{array}{c} F_{1n}=\frac{2\times N_{n}}{\sum N+\sum n}, \end{array}$$

where *N* is the total number of normal signals recognized by the algorithm, *N*_*n*_ is the number of correct signals classified as normal by the algorithm, and *n* is the total number of normal signals.

(9) $$\begin{array}{c} F_{1o}=\frac{2\times O_{o}}{\sum O+\sum o}, \end{array}$$

where *O* is the total number of signals identified by the algorithm as “other,” *O*_*o*_ is the correct number of signals classified by the algorithm as “other,” and *o* is the total number of “other” signals.

(10) $$\begin{array}{c} F_{1p}=\frac{2\times P_{p}}{\sum P+\sum p}, \end{array}$$

where *P* is the total number of noise signals recognized by the algorithm, *P*_*p*_ is the correct number of noise signals classified by the algorithm, and *p* is the total number of noise signals.

(11) $$\begin{array}{c} F_{\text{overall}}=\frac{\left(F_{1n}+F_{1a}+F_{1o}\right)}{3}. \end{array}$$

Because the noise signals are too small and unbalanced, the result of the entire dataset is unstable, and the first three types of signals are selected as the final F1 index. Even so, the F1 score of noise will also affect the other three types. In addition to F1, we also use true positive (TP), true negative (TN), false positive (FP), and false negative (FN) to calculate accuracy (Acc), specificity (Spe), and sensitivity (Sen). The calculation formula is as follows:

(12) $$\begin{array}{c} \text{Acc}=\frac{\text{TP}+\text{TN}}{\text{TP}+\text{TN}+\text{FP}+\text{FN}},\\ \text{Spe}=\frac{\text{TN}}{\text{TN}+\text{FP}},\\ \text{Sen}=\frac{\text{TP}}{\text{TP}+\text{FN}}. \end{array}$$

## 5. Results

Four experiments are used to verify the feasibility and efficiency of the proposed feature fusion model. The first three experiments are comparative experiments.

### 5.1. Experiments Based on Single Feature

#### 5.1.1. Experiments Based on Traditional Feature

In this experiment, after the ECG signal is denoised, its statistical features and frequency domain features are extracted manually based on expert knowledge, and finally, the XGBoost (Extreme Gradient Boosting) classifier is used for classification. The experimental block diagram based on traditional feature extraction and classification is shown in Figure 9.

The XGBoost parameters are tuned using random grid search cross-validation, and the optimal parameters are selected. The minimum leaf node weight is set to 20, the maximum depth of the tree is set to 11, the subsample is set to 0.8, the colsample_bytree is set to 0.9, the learning rate is 0.2, and the maximum depth of the tree is 11.

The minimum loss function is reduced to 1, the softmax objective function is used for classification, and the final F1 is 75%.

#### 5.1.2. Experiments Based on Deep Learning Feature

In this experiment, the ECG signal is detected based on the model of residual network and gated recurrent unit. The experimental block diagram of using deep learning feature extraction to classify atrial fibrillation is shown in Figure 10.

Firstly, padding the original ECG data. Since the central electrical data of the database varies from 9 s to 61 s and the convolutional network requires equal length input, the ECG data is padded the same length. This paper uses the maximum length of the ECG signal. The sampling rate is 300 Hz, and the calculated maximum length is 18286. Each ECG data is inputted into the residual network. The residual network includes six residual convolution blocks, and each of them consists of a convolution block, a residual block, and a one-dimensional average pooling layer. Each convolutional block includes four parts: a one-dimensional convolution layer with a step size of 1, a batch normalization layer, a linear unit with leakage correction, and a spatial random inactivation layer. After the residual network, data is inputted to the gated recurrent unit for training. The number of neurons in the gated recurrent unit is 32. Finally, it is output through the fully connected layer. F1 ended up at 83%.

### 5.2. Experiments Based on Feature Concatenation Fusion

In this experiment, the features are simply spliced and fused and input to the fully connected layer for classification.

The feature vectors based on expert knowledge and the feature vectors extracted by the residual network and gated recurrent unit are spliced in series to obtain the fused features and input to the fully connected layer for classification. The specific process is as follows: firstly, add a flatten layer to make the traditional feature vector one-dimensional; then, use the deep learning model for training, the output of the last hidden layer of the recurrent unit as the deep learning feature vectors; finally, use the concatenation method to integrate the two feature vectors into one, and add a fully connected layer for classification. The value of F1 is 85%, and the accuracy and loss diagrams are shown in Figures 11 and 12.

### 5.3. Experiments Based on DCCA Feature Fusion

In this experiment, the feature vectors extracted by the traditional feature extraction method based on expert knowledge and the deep learning feature vectors extracted using the gated recurrent unit and residual network are fused with discriminant canonical correlation analysis and then input to the fully connected layer for feature classification. The final accuracy on the verification set is 91.7, and F1 is 88%. The accuracy and loss diagrams are shown in Figures 13 and 14. From Table 2, it can be seen that the DCCA-based fusion method is better than the concatenation fusion method. Compared with simple concatenation fusion, the DCCA method considers the correlation among samples and the category information of the sample, which contains less redundant information than the series fusion method.

As can be seen from Table 2 and Figure 12, that compared to using single feature, the method of feature fusion for AF signal detection can obtain better classification accuracy. Compared with single feature extraction, the F1 score is increased by 2% when using simple feature fusion, and compared with the simple feature fusion method, the F1 score is increased by 3% when using DCCA feature fusion.

### 5.4. Experimental Comparative Analysis

In order to verify the effectiveness of the proposed method, comparisons are also performed with previous studies.  Table 3 lists some of the published ECG signal detection research results based on the same dataset, which includes traditional feature extraction, machine learning based on expert knowledge, and deep learning-based methods. It can be seen from Table 3 that the use of a single method requires complex preprocessing, and the final F1 value is 79.4%, which is not ideal [24]. The signal detection model using the expert knowledge feature extraction algorithm has better interpretability. On the other hand, deep neural networks are used to autonomously learn features from ECG records. The conventional method is very easy to learn. Xiong et al. [25] proposed a 16-layer deep convolutional neural network for the automatic classification of ECG signal, the final F1 is 82.0%, and the accuracy is 80.2%. The feature fusion method based on discriminative canonical correlation analysis proposed in this paper can fuse the advantages of the two and achieve a more ideal result. The F1 value is 88%. The accuracy, sensitivity, and specificity are 91.7%, 90.4%, and 93.2%, respectively, conducive to more accurate ECG signal detection. It is foreseeable that with the further accumulation of datasets, the feature fusion model can achieve more powerful classification capabilities.

## 6. Conclusion

This paper proposes a classification method for atrial fibrillation signals based on the feature fusion of discriminant canonical correlation analysis. This method can not only extract the deep learning features of ECG signals but also fuse the traditional features of ECG signal samples. With DCCA, the maximum and minimum correlations among classes of different sample types are considered, and the recognition results are better than that of series feature fusion as well as the use of deep learning or traditional features alone. This method has been verified on the public short single-lead ECG dataset of the 2017 PhysioNet/CinC Challenge, with a verification accuracy of 91.7%, a sensitivity of 90.4%, and a specificity of 93.2%. The database used in this article itself has the problem of large differences among various categories, which shows that the fusion method in this article improves the overall accuracy while taking into account other measurement standards, and steadily improves the classification performance of ECG signals. However, this paper only considers the comprehensive and complementary representation of ECG features through feature-level fusion and does not consider the fusion of decision-making layers, such as neural network algorithms, hidden Markov models, and combinations of multiple classifiers. In future researches, the classification model and feature fusion method will be further improved. On the basis of DCCA feature fusion technology, core-based DCCA will be introduced. At the same time, more cutting-edge classifiers will be selected for classification and recognition, which will be more effective to improve recognition results.

## Figures and Tables

**Figure 1:** Deep learning feature extraction uses ResNet (residual network) and GRU (gated recurrent unit).

**Figure 2:** ECG detection algorithm detects QRS.

**Figure 3:** RR intervals and P waves [32].

**Figure 4:** The structure of the proposed simple feature fusion.

**Figure 5:** The specific process of simple feature fusion.

**Figure 6:** The structure of the proposed DCCA feature fusion.

**Figure 7:** A graphical representation of the relationship between sample characteristics. Among them, hexagon and circle represent each feature, solid line represents the correlation within the class, and dashed line represents the correlation between classes.

**Figure 8:** Block diagram for realizing canonical correlation analysis.

**Figure 9:** Block diagram of AF by traditional feature experimental pipeline.

**Figure 10:** Block diagram of AF by deep learning feature experimental pipeline.

**Figure 11:** The accuracy diagram of series feature fusion.

**Figure 12:** The loss diagram of series feature fusion.

**Figure 13:** The accuracy diagram of DCCA feature fusion.

**Figure 14:** The loss diagram of DCCA feature fusion.

**Table 1:** The PhysioNet 2017 dataset.

Type	Recording	Average time length (s)
Normal	5076	31.9
AF	758	31.6
Other rhythm	2415	34.1
Noisy	279	27.1

**Table 2:** The result of the different model.

Model	*F*_1*n*_	*F*_1*a*_	*F*_1*o*_	*F*_overall_	Acc	Spe	Sen
Expert features	87%	73%	65%	75%	79%	82%	72%
Resnet+GRU	91%	81%	77%	83%	86%	85%	84%
Simple fusion	92%	83%	80%	85%	88%	89%	86%
Proposed	93%	88%	84%	88%	92%	93%	90%

**Table 3:** Comparison of previous studies of ECG based on the PhysioNet/CinC challenge 2017 public dataset.

Method	*F*_1*n*_	*F*_1*a*_	*F*_1*o*_	*F*_overall_	Acc	Spe	Sen
Convolutional recurrent neural network [23]	92.4%	81.4%	80.9%	84.9%	87.5%	94.6%	82.9%
Decision tree ensemble [24]	88.9%	79.1%	70.2%	79.4%	——	——	——
16-layer 1D residual convolutional network [25]	90.0%	82.0%	75.0%	82.0%	80.2%	——	——
2D convolutional network with LSTM layer [26]	88.8%	76.4%	72.6%	79.2%	82.3%	——	——
1DCNN containing residual blocks and recurrent layers [27]	91.9%	85.8%	81.6%	86.4%	——	——	——
Proposed in this paper	93.1%	88.3%	84.0%	88.3%	91.7%	93.2%	90.4%%

## Data Availability

The datasets used during the present study are available from the corresponding author upon reasonable request or can be downloaded from https://www.physionet.org/content/challenge-2017/1.0.0/.
